# Oxidative Stress Mediated Cytotoxicity, Cell Cycle Arrest, and Apoptosis Induced by *Rosa damascena* in Human Cervical Cancer HeLa Cells

**DOI:** 10.1155/2021/6695634

**Published:** 2021-01-28

**Authors:** Mai M. Al-Oqail, Nida N. Farshori, Ebtesam S. Al-Sheddi, Shaza M. Al-Massarani, Quaiser Saquib, Maqsood A. Siddiqui, Abdulaziz A. Al-Khedhairy

**Affiliations:** ^1^Department of Pharmacognosy, College of Pharmacy, King Saud University, Riyadh 11495, Saudi Arabia; ^2^DNA Research Chair, Zoology Department, College of Science, King Saud University, P.O. Box 2455, Riyadh 11451, Saudi Arabia; ^3^Zoology Department, College of Science, King Saud University, P.O. Box 2455, Riyadh 11451, Saudi Arabia

## Abstract

*Rosa damascena* Mill (Damask rose), belonging to the Rosaceae family, is known for medicinal purposes in traditional medicine system. However, its anticancer activity has not been studied yet in detail. Herein, we aimed to investigate the cytotoxic effects of *R. damascena* hexane (RA-HE) and methanolic (RA-ME) extracts against human breast (MCF-7), lung epithelial (A-549), and cervical (HeLa) cancer cells. The RA-HE and RA-ME showed more potent cytotoxic effects against HeLa cells with an IC_50_ of 819.6 and 198.4 *μ*g/ml, respectively. Further, cytotoxic concentrations of most effective extract (RA-ME) were used to evaluate the mechanism of cytotoxicity involved in HeLa cells. A concentration-dependent induction of lipid peroxidation (LPO) and reduction of glutathione (GSH) in HeLa cells treated with 250-1000 *μ*g/ml of RA-ME confirms the association of oxidative stress. We also detected a noteworthy increase in reactive oxygen species (ROS) production and a decline in mitochondrial membrane potential (MMP) level in RA-ME-exposed HeLa cells. Flow cytometric data showed a strong dose-response relationship in cell cycle analysis between subG1 phase in HeLa cells and RA-ME treatment. Similarly, a concentration-dependent increase was recorded with Annexin V assay in HeLa cells going to late apoptosis. In conclusion, our findings suggest that RA-ME-induced cytotoxicity and apoptosis in HeLa cells are mediated by oxidative stress.

## 1. Introduction

Cancer is the second leading cause of the mortality worldwide and is main health problem globally because of the uncontrolled cell growth [1]. Cancer elaborates uncontrolled growth of normal cells triggered by genetic changes and variabilities, subsequent in the production of malignant cells, and initial of development of secondary malignant growths [2]. These genetic changes could be due to the exposure of pesticides, smoking, absorption of carcinogenic chemicals, or alterations in the immune system and hormonal balance [3]. As cancer is typically detected at an advanced stage, the diagnosis is poor and treatment is mainly unsuccessful [4]. The deficiency in early detection and lack of effective therapeutic agents are the foremost causes of poor cancer control and diagnosis [5]. The treatment of cancer includes chemotherapy, surgery, and/or radiation. Various chemotherapeutic agents often used have been found to be less effective and are associated with severe side effects such as damage to normal cells [6]. Hence, the search for alternative therapeutic effective agent with less side effects is needed. Globally, after breast and colon cancer, cervical cancer is the third leading malignancy among women [7]. Cervical cancer is one of the most common cancers in female living in middle- and low-income countries [8]. Although incidence and death rates have been declined in past decades, but due to the population aging, the number of new cases and mortality has increased by 0.5%/year [9]. Because of population and aging, estimated number of new cases is expected to increase by 2025, if incidents remain the same at 2002 [10]. Further, in order to broadly report this serious health problem, initial recognition and medicine with clinical efficacy are to be required. The field of natural product research has become one of the most interesting subjects in the advancement of novel therapeutic agents [11]. Plants have played a leading role in the old system of remedy with particularly elongated history in the treatment of cancer diseases [12]. A number of plant extracts such as *cotinus coggygria* [13], *Aristolochia ringens* [14], *Tabernaemontana divaricate* [15], and *Artemisia annua* [16] have been reported to possess cytotoxic effects against HeLa cells. The earlier studies have demonstrated that the cytotoxic phytochemicals are capable to induce apoptosis/necrosis by obstructing different signaling pathways, which leads to cell cycle arrest and cell death [17]. Cancer cells have several molecular mechanisms to improve and suppress apoptosis that plays key role in cancer development [18]. Therefore, induction in apoptosis/necrosis by cytotoxic agents can be a fundamental beneficial method towards cancer chemotherapy [19]. *Rosa damascena* Mill L (Damask rose), known as Gole Mohammadi, is one of the most important species of Rosaceae family. *R. damascena*, an ornamental plant, is primarily cultivated for the use in food industries and perfumes [20]. Apart from these, this plant is also being used for medicinal purposes in traditional medicine system [21]. A number of products and isolated constituents from seeds, flowers, and petals of *R. damascena* have been studied in different *in vivo* and *in vitro* model systems [22]. The beneficial effects of *R. damascena* extracts have been established for the management of menstrual bleeding and digestive problem [23], cough [24], gentle laxative [25], analgesic [26], brain function [27], and cardiovascular function [28]. The antioxidant [29], antimicrobial [30], anti-HIV [31], antidiabetic [32], antiageing [33], and anti-inflammatory [34] activities of *R. damascena* have also been well-documented. There are few reports that reveal that *R. damascena* extracts and oils induced cytotoxic effects against various cancer cell lines [35–38]. In another study, the cytotoxic potential of the leaf bud and flower extracts of *Crataegus microphylla* plant of Rosaceae family against HeLa cells have also been reported [39]. But there has been only limited investigation on the cytotoxic effects of *R. damascena*; however, detailed mechanistic studies have not been conducted yet. Therefore, this study was conducted to investigate the mechanism(s) of cytotoxicity induced by *R. damascena* against three different carcinoma cell lines, i.e., human breast (MCF-7), human lung epithelial (A-549), and human cervical (HeLa). In this study, firstly, we screened the cytotoxicity of hexane (RA-HE) and methanolic (RA-ME) extracts of *R. damascena* using MTT assay, neutral red uptake assay, and morphological changes. Secondly, the cytotoxic concentrations of most effective extract were used to evaluate the mechanism involved in the cytotoxicity against sensitive cancer cells, HeLa.

## 2. Material and Methods

### 2.1. Chemicals and Culture Medium

Cell culture medium (DMEM) with high glucose, sodium bicarbonate, MTT, neutral red, Rhodamine (Rh123), and 2′,7′-dichlorofluorescin (DCF-DA) dye was procured from Sigma Aldrich, USA. Fetal bovine serum (FBS), antibiotic-antimycotic (100x solution) (Cat. No. 15240-062, Gibco), and trypsin were procured from Gibco, Life Technologies, USA. Flow cytometric kits were purchased from Backman Coulter, USA. All other specified chemicals and reagents were obtained from Sigma Aldrich, USA, unless indicated otherwise.

### 2.2. Cell Culture

Human breast adenocarcinoma (MCF-7), human lung epithelial (A-549), and human cervical carcinoma (HeLa) cell lines were obtained from American Type Culture Collection (ATCC), USA. The cell lines were grown in DMEM with 10% FBS and 1% antibiotic solution. All cell lines were maintained in 25 cm^2^ flasks at 37°C in a humidified atmosphere containing 5% CO_2_.

### 2.3. Plant Collection and Extractions

The fresh *R. damascena* flowers were collected from a rose farm, Taif, Saudi Arabia. The roses were cut into small pieces, air-dried under shade at 25°C, and converted into a course powder. The extraction was done by maceration. Briefly, 10 g of powdered *R. damascena* was extracted with hexane and methanol, respectively. Then, the filtrate was collected in a beaker by filtration and dried at 40°C in a rotary evaporator. The extracts were separately obtained, and the dried hexane extract was named as RA-HE and methanolic extract as RA-ME. Both the extracts were stored at 4°C until further use. The extracts were diluted in dimethyl sulfoxide (DMSO) for bioassays. The final concentration of DMSO used in the assays was 0.02%.

### 2.4. Cytotoxicity Experiments

The *in vitro* cytotoxicity of RA-HE and RA-ME against MCF-7, A-549, and HeLa cells was determined by MTT, neutral red uptake, and cell morphology assays [40].

### 2.5. MTT Assay

Briefly, cells were seeded into a 96-well culture plate at 1 × 10^4^ cells in each well. Cells were then exposed to varying concentrations (0-1000 *μ*g/ml) of RA-HE and RA-ME. The plates were placed in a humidified 5% CO_2_ incubator for 24 h. Then, MTT solution (10 *μ*l of 5 mg/ml MTT stock) was added to each well and incubated for 4 h. The colored formazan crystal formed was dissolved in dimethyl sulfoxide. Finally, absorbance was measured at 550 nm using microplate reader [40].

### 2.6. NRU Assay

Following the protocol [40], the NRU assay was performed. In brief, all the cells were plated in a 96-well plate at a density of 10,000 cells/well. Then, cells were exposed to varying concentrations (0-1000 *μ*g/ml) of RA-HE and RA-ME for 24 h. The cells were then incubated for 3 h in a medium supplemented with 50 *μ*g/ml of NR dye. After incubation, the plates were washed and dye was extracted in ethanol: acetic acid: water (50 : 1 : 49). Finally, absorbance was measured at 550 nm using microplate reader. All the assays were performed in replicates for each RA-HE and RA-ME concentrations. Three replicates were examined in each experiment. The percent cell viability was calculated as follows:

(1) $$\begin{array}{c} \%\text{survival}=\text{mean experimental absorbance}/\text{mean control absorbance}\times 100. \end{array}$$

### 2.7. Morphology Assay

To analyze the cell morphology induced by RA-HE and RA-ME in MCF-7, A-549, and HeLa cells, 1 × 10^4^ cells were seeded into a 96-well culture plate. After 24 h of exposure, alterations in the cellular morphology were observed at 20x magnification using a light microscope (Olympus, CKX41, Japan).

### 2.8. Oxidative Stress Measurements by LPO and GSH

To measure the LPO and GSH content, HeLa cells were plated in 6-well plates at 1 × 10^5^ cells in every well. The cells were then exposed to 250, 500, and 1000 *μ*g/ml of RA-ME for 24 h. After treatment, control and treated cells were harvested and sonicated and total protein was measured by Lowry et al. [41]. The LPO content in HeLa cells was measured by TBARS (thiobarbituric acid-reactive substance) method [42], and GSH content was measured according to the method of Chandra et al. [43].

### 2.9. Reactive Oxygen Species (ROS) Measurements

The intracellular ROS level in HeLa cells was determined by DCF-DA fluorescence dye following the method described earlier [44]. Briefly, HeLa cells were seeded into 24-well plates with a density of 2 × 10^4^ cells/well in complete medium. Then, cells were exposed to 250-1000 *μ*g/ml of RA-ME for 24 h. After that, cells were rinsed with PBS and then incubated with 20 *μ*M of DCF-DA dye in dark for 1 h. The qualitative ROS level was examined under the microscope, and qualitative fluorescence of cells was measured by fluorescent reader at 485/530 nm excitation/emission (Fluoroskan Ascent, Thermo-Scientific, Finland).

### 2.10. Mitochondrial Membrane Potential (MMP) Analysis

Rhodamine 123-based fluorescence measurement was used to analyze the alterations of MMP in HeLa cells after the exposure of RA-ME using the method [44]. Briefly, HeLa cells were plated in 24-well plates with a density of 2 × 10^4^ cells in each well. Then, cells were treated with 250-1000 *μ*g/ml of RA-ME for 24 h. After that, cells were incubated with 10 *μ*g/ml of Rh123 dye for 60 min in the dark and fluorescence of MMP was analyzed under fluorescence microscope. The quantitative measurements of MMP in HeLa cells were done by measuring the plate at 485/530 nm excitation/emission.

### 2.11. Cell Cycle Analysis

To analyze the cell cycle arrest induced by RA-ME, HeLa cells (5 × 10^4^ cells/well) were seeded in 24-well culture. Cells were then exposed to 250-1000 *μ*g/ml of RA-ME for 24 h. After treatment, cells were rinsed with PBS and fixed in 70% cold ethanol for 1 h. Further, cells were rinsed and dispersed in a staining solution containing 50 *μ*g/ml propidium iodide (PI) and 50 *μ*g/ml RNase A. After incubating at room temperature for 1 h, distribution of cells in each phase of cell arrest was examined by PI staining using Beckman Coulter Epics XL-MCL flow cytometer.

### 2.12. Apoptosis Assay

Apoptosis analysis in HeLa after the exposure of RA-ME was performed using commercially available Annexin V-PI apoptosis kit (Beckman Coulter, USA). Briefly, HeLa cells were plated in culture plate and treated with 0, 250, 500, and 1000 *μ*g/ml of RA-ME for 24 h. After treatment, cells were collected and washed with chilled PBS. After centrifugation, the cell pellet of control and exposed cells was resuspended in 1× binding buffer containing 10 *μ*l of each Annexin V and PI for 20 min in the dark. The distribution of apoptosis/necrosis cells was recorded by using flow cytometer (Beckman Coulter Epics XL-MCL).

### 2.13. Statistical Analysis

The data analysis was done by one-way analysis of variance (ANOVA) using Dunnett's test. The level of statistical analysis selected was *p* < 0.05 unless indicated otherwise. Results were expressed as mean ± SD obtained from three independent experiments.

## 3. Results and Discussion

### 3.1. Cytotoxicity

The cell viability of three carcinoma cell lines, MCF-7, A-549, and HeLa, was assessed by MTT and NRU assays after the exposure of RA-HE and RA-ME at 0-1000 *μ*g/ml for 24 h. The results showed that all the cell lines responded to cytotoxic effects of RA-ME in a concentration dependent manner (Figure 1). However, RA-HE has not shown cytotoxic effects on MCF-7 and A-549 cells and less cytotoxic effects on HeLa cells in contrast to RA-ME. RA-ME at 500 and 1000 *μ*g/ml significantly decreased the viability of MCF-7 and A-549 cells. The cell viability was recorded as 81% and 70% in MCF-7 and 72% and 48% in A-549 cells, respectively, at 500 and 1000 *μ*g/ml of RA-ME. However, a significant reduction in the viability of HeLa cells was recorded even at 100 *μ*g/ml and above concentrations. The cell viability was recorded as 71%, 37%, 25%, and 13% at 100, 250, 500, and 1000 *μ*g/ml of RA-ME, respectively. The RA-HE was also found to reduce the cell viability of HeLa cells up to 75% and 39% at 500 and 1000 *μ*g/ml, respectively. NRU assays also revealed similar kind of cytotoxic response of RA-HE and RA-ME against MCF-7, A-459, and HeLa cells. The results showed that RA-ME reduced the viability of all three cells in a concentration-dependent manner (Figure 2). The viability of cells was found to be 83% and 72% in MCF-7, 70% and 45% in A-549, and 27% and 15%, respectively, at 500 and 1000 *μ*g/ml of RA-ME. However, RA-HE was found to be noncytotoxic to MCF-7 and A-549 cells, but the viability was reduced to 73% and 42% in HeLa cells at 500 and 1000 *μ*g/ml. In contrast, RA-HE and RA-ME were found to induce cytotoxicity only in HeLa cell line, but RA-HE showed slightly less cytotoxic effects to HeLa cells even at higher concentrations compared to RA-ME. Therefore, RA-ME was chosen for further analysis in HeLa cells. The half maximal inhibitory concentration (IC_50_) values of RA-HE and RA-ME obtained on MCF-7, A-549, and HeLa cells are presented in Table 1. These findings were also substantiated by morphological observations. As shown in Figure 3, RA-ME decreased the maximum density of HeLa cells compared to MCF-7 and A-549 cells. In this study, we used MTT and NRU assays to assess the cytotoxic potential of RA-HE and RA-ME in MCF-7, A-549, and HeLa cells. These assays are routinely being used to screen the cytotoxic potential of plant extract against cancer cell lines [45]. The live cells reduced yellow MTT to purple formazan crystal by mitochondrial dehydrogenase enzyme [46]. Neutral red is a weak cationic weak dye which accumulates in lysosome of living cells but not in dead cells by nonionic passive diffusion [47]. The amount of dye taken up by cells is assumed to be relative to the total number of live cells present. Our results showed that MTT and NRU assays revealed a concentration-dependent cytotoxicity of RA-HE and RA-ME against cancer cell lines. The results showed that RA-ME at 100 *μ*g/ml and above concentrations inhibits the cell viability of HeLa cells. Our results are consistent with previous reports showing that alcoholic extracts of *Rosa damascena* induced cytotoxic effects against HeLa cell line in the range of 100-1000 *μ*g/ml concentrations [36]. In our study, methanolic extract of R. *damascena* (RA-ME) showed highest cytotoxic response in HeLa cell line with IC_50_~200 *μ*g/ml, which is consistent with Artun et al. [13], who have shown that methanolic extract of *R. damascena* exhibited cytotoxicity effects on HeLa cells with IC_50_ of 265 *μ*g/ml. Other reports have also showed cytotoxic activities of *Rosa damascena* and its ingredients against human prostate, lung, and breast cancer cell lines [35]. Hagag et al. [48] have also shown that *Rosa damascena* exhibited anticancer potential against MCF-7 and HepG2 cells.

### 3.2. Oxidative Stress Measurements by LPO and GSH

Oxidative stress is well-known to be associated with the molecular mechanism of bioactive constitutes induced apoptosis and cytotoxicity [49]. To study the role of oxidative stress in RA-ME-induced HeLa cell death, we have performed the LPO and GSH assays (Figure 4). Our results obtained from LPO assay exhibited a significant dose-dependent increase in the LPO in RA-ME-exposed HeLa cells. A 35%, 55%, and 93% enhancement in LPO in HeLa cells was recorded at 250, 500, and 1000 *μ*g/ml of RA-ME, respectively (Figure 4(a)). Our results clearly showed that RA-ME significantly induced the LPO level in HeLa cells. Many studies have also shown that plant extracts exhibited oxidative stress-mediated cancer cell death by increasing the LPO and decreasing the GSH activities [50, 51]. GSH plays a significant part in the defense of cells on oxidative stress [52]. It has also been documented that cellular GSH level is an important component for the activity of anticancer agents [53]. In this study, we found that GSH level was significantly reduced in RA-ME-treated HeLa cells. A maximum reduction of 64% was observed at 1000 *μ*g/ml of RA-ME followed by 30% and 8% at 500 and 250 *μ*g/ml of RA-ME as compared to untreated control (Figure 4(b)). The depletion in GSH content in HeLa cells could be resulted due to the increased intercellular oxidation of GSH or inhibition of GSH synthesis by the plant extract. These findings suggest that reduction in GSH level by RA-ME may contribute to increase of ROS generation in the cells producing redox imbalance which leads to oxidation of biomolecules causing cell death. Similarly, Wageesha et al. [54] reported that treatment of HeLa cells with “Le Pana Guniya” (LPG), a well-known anticancer herbal medicine, caused depletion in GSH level.

### 3.3. ROS Measurement

The increase ROS production has been reported as one of the major causes of apoptosis in cancer cells and has been recognized into a promising therapeutic approach for the cancer treatments [55]. Herein, we have measured the quantitative and qualitative ROS production in HeLa cells exposed to cytotoxic concentrations of RA-ME. As shown in Figure 5(a), RA-ME significantly induced ROS generation in HeLa cells as examined by fluorescence microscope. An increase of 29%, 68%, and 101% in ROS generation was observed at 250, 500, and 1000 *μ*g/ml, respectively, in HeLa cells exposed to RA-ME for 24 h as measured by using fluorescence spectrophotometer (Figure 5(b)). Based on obtained data showing an increase in ROS generation indicated that RA-ME-induced cytotoxicity and apoptosis in HeLa cells are mediated through ROS generation. The increase level of ROS production has also been reported to be involved in the process of anticancer mechanism of potential anticancer drugs [56] and plant extract-induced apoptosis in human prostate (CA-2B), human breast (MCF-7), and human lung (PC-9) cancer cells [57].

### 3.4. MMP Analysis

Depolarization in MMP is known as one of the properties of apoptosis progression in cells [58]. To confirm this process, we measured the mitochondrial membrane potential in HeLa cells. The cells were exposed to RA-ME at 250-1000 *μ*g/ml for 24 h. As given in Figure 6, the florescence images revealed a concentration-dependent decrease in MMP (Figure 6(a)). The quantitative data also exhibited that RA-ME decreased the MMP by 16%, 38%, and 71% at 250, 500, and 1000 *μ*g/ml, respectively (Figure 6(b)). As observed here, a decrease in the intensity of dye which indicated a disruption of MMP suggests that the HeLa cell death induced by RA-ME is mitochondrial dependent. The cytotoxicity and apoptosis responses through disruption of MMP in other cancer cells have also been investigated [59]. Numerous studies also revealed the apoptotic possessions of Rosa species, such *Rosa canina* extract in human colon cancer [60] and human lung and prostate cancer cells [61] through depolarization in mitochondrial membrane potential.

### 3.5. Cell Cycle Analysis

The cell cycle arrest in HeLa cells treated with *R. damascena* extract (RA-ME) was analyzed by flow cytometer. As shown in Figure 7, there was a strong dose-response relationship between subG1 phase in HeLa cells and RA-ME treatment. All the concentrations of RA-ME used significantly increased the cell numbers in subG1 phase (apoptosis cells). After 24 h of treatment, percentages of cells in subG1 phase were 4.21%, 74%, 84.6%, and 88.6% in control in 250, 500, and 1000 *μ*g/ml of RA-ME, respectively (Figures 7(a)–7(d)). Our results showed that RA-ME induced a dose-dependent accumulation of cells in G1 phase. Consistent with our results, Kilinc et al. [61] in *Rosa canina* extract arrested cell cycle of human lung and human prostate cancer cells in subG1/G0 phase. Similarly, one of the main components of Rose, Geraniol-treated pancreatic cancer cells, has also exhibited dose-dependent increases in the percentage of cells in subG1/G0 phase of cell cycle and decreases the cells present in G2/M phases [62].

### 3.6. Apoptosis Assay

To investigate the apoptotic effects of *R. damascena* extract (RA-ME) on HeLa cells, the flow cytometric analysis was performed. Apoptosis analysis was done using Annexin V-PI apoptosis assay. As shown in Figures 8(a)–8(d), a dose-dependent increase in the percentage of late apoptosis (quadrant 2) cells was found in HeLa cells. The percentages of apoptosis cells in untreated control and RA-ME-treated cells (quadrant 2) were 1.21%, 59.3%, 81.3%, and 88.9% in 0, 250, 500, and 1000 *μ*g/ml, respectively (Figures 8(a)–8(d)). Our results showed that RA-ME induces cellular apoptosis in human cervical cancer (HeLa) cells with the increasing concentrations. These apoptosis cells show an increase expression of Annexin V positive cells in RA-ME-exposed HeLa cells compared to control. The maximum apoptosis cells were found at 1000 *μ*g/ml of RA-ME. Our results are also supported by Khatib et al. [63], who have shown that *R. damascena* oil induced cytotoxicity in gastric cancer cell line (MKN45) through apoptosis mechanism. Turan et al. [60] have also demonstrated that *Rosa canina* extract exhibits concentration-dependent cytotoxic effects against human colon cancer cells by inducing apoptosis. Induction in cancer cell apoptosis has been extensively studied, making it an important indicator for the development of anticancer agents [55]. Earlier reports have also demonstrated that cytotoxic phytochemicals either induced apoptosis or block the signaling pathways, thus leading to cell cycle arrest or cell death [64]. Cancer cells are known to possess molecular mechanism that alleviates apoptosis which plays an important role in the progression of cancer [19]. Therefore, induction in apoptosis induced by cytotoxic agents can be an essential therapeutic method in the direction of cancer chemotherapy.

## 4. Conclusions

In conclusion, the present study demonstrated the mechanism of *R. damascena* against cancer cells *in vitro*. Our findings revealed that RA-ME-induced apoptosis and cytotoxicity in HeLa cells are associated with oxidative stress formation, ROS production, mitochondrial depolarization, and cell cycle arrest. Based on results obtained in the present investigation, we can assume that the cell death induced by RA-ME in HeLa cells is due to the oxidative stress. The cytotoxic effects of *R. damascena* observed in this study provide a detail insight knowledge on it. However, further studies are required to understand specific mechanism(s) involved in *R. damascena*-induced cancer cell death.

## Figures and Tables

**Figure 1:** Cytotoxic potential of (a) RA-HE and (b) RA-ME against human breast (MCF-7), human lung (A-549), and human cervical (HeLa) carcinoma cell lines. MCF-7, HeLa, and A-549 cells were treated with increasing concentrations (0-1000 *μ*g/ml) of RA-HE and RA-ME for 24 h. Cell viability was determined by MTT assay. Each diagram represents as mean ± SD of three experiments. Significant difference ^∗^*p* < 0.5 and ^∗∗^*p* < 0.01 from the control.

**Figure 2:** Cytotoxic potential of (a) RA-HE and (b) RA-ME against human breast (MCF-7), human lung (A-549), and human cervical (HeLa) carcinoma cell lines. MCF-7, HeLa, and A-549 cells were treated with increasing concentrations (0-1000 *μ*g/ml) of RA-HE and RA-ME for 24 h. Cell viability was determined by neutral red uptake (NRU) assay. Each diagram represents as mean ± SD of three experiments. Significant difference ^∗^*p* < 0.5 and ^∗∗^*p* < 0.01 from the control.

**Figure 3:** Representative light microscopy images of MCF-7, A-549 cells, and HeLa treated with their higher concentration, i.e., 1000 *μ*g/ml for 24 h. The images were taken with magnification of 20x.

**Figure 4:** RA-ME-induced oxidative stress in human cervical carcinoma (HeLa) cells. The cells were treated with increasing concentrations (0-1000 *μ*g/ml) of RA-ME for 24 h. (a) Percent increase in lipid peroxidation (LPO) level and (b) depletion in glutathione (GSH) level. Significant difference ^∗^*p* < 0.5 and ^∗∗^*p* < 0.01 from the control.

**Figure 5:** (a) Green fluorescence staining using DCF-DA dye showing ROS generation in HeLa cells. Cells were treated with 250-1000 *μ*g/ml of RA-ME for 24 h. (b) Bar diagram showing percent induction in ROS generation. Significant difference ^∗^*p* < 0.5 and ^∗∗^*p* < 0.01 from the control.

**Figure 6:** (a) Mitochondrial membrane potential (MMP) staining using Rhodamine 123 in control and treated HeLa cells with RA-ME. Cells were exposed to 250, 500, and 1000 *μ*g/ml of RA-ME for 24 h. (b) Bar diagram showing percent change in decreased mitochondrial membrane potential. Significant difference ^∗^*p* < 0.5 and ^∗∗^*p* < 0.01 from the control.

**Figure 7:** Flow cytometric images presenting cell cycle arrest in HeLa cells treated with RA-ME at 250, 500, and 1000 *μ*g/ml for 24 h. The images showing an increase in subG1 peak with the increasing doses of RA-ME.

**Figure 8:** Representative flow cytometry analysis results obtained from Annexin V-FITC/PI assay. The HeLa cells were exposed to RA-ME at 250, 500, and 1000 *μ*g/ml for 24 h. Percentage of early apoptotic, late apoptotic, and necrotic cells are shown by the scatter plots.

**Table 1:** Inhibitory concentration (IC_50_) of the RA-HE and RA-ME on MCF-7, A-549, and HeLa cell lines.

Cell lines	IC_50_ (*μ*g/ml)	
	RA-HE	RA-ME
MCF-7	>1000	>1000
A-549	>1000	961.5
HeLa	819.6	198.4

## Data Availability

The data used to support the findings of this study are included within the article.

## References

[1] Nagai H., Kim Y. H. (2017). Cancer prevention from the perspective of global cancer burden patterns. *Journal of Thoracic Disease*.

[2] Mazumder K., Biswas B., Raja I. M., Fukase K. (2020). A review of cytotoxic plants of the Indian subcontinent and a broad-spectrum analysis of their bioactive compounds. *Molecules*.

[3] Kaur K., Kaur R. (2018). Occupational pesticide exposure, impaired DNA repair, and diseases. *Indian Journal of Occupational and Environmental Medicine*.

[4] Caplan L. (2014). Delay in breast cancer: implications for stage at diagnosis and survival. *Frontiers in Public Health*.

[5] Bratulic S., Gatto F., Nielsen J. (2019). The Translational Status of Cancer Liquid Biopsies. *Regenerative Engineering and Translational Medicine*.

[6] Johnstone R. W., Ruefli A. A., Lowe S. W. (2002). Apoptosis: a link between cancer genetics and chemotherapy. *Cell*.

[7] Ferlay J., Soerjomataram I., Ervik M. (2013). *GLOBOCAN 2012 v1.0, Cancer Incidence and Mortality Worldwide: IARC CancerBase No. 11. International Agency for Research on Cancer*.

[8] Arbyn M., Castellsagué X., de Sanjosé S. (2011). Worldwide burden of cervical cancer in 2008. *Annals of Oncology*.

[9] Denny L., Herrero R., Levin C., Kim J. J., Gelband H., Jha P., Sankaranarayanan R., Horton S. (2015). Cervical cancer. *Disease control priorities*.

[10] Parkin D. M., Almonte M., Bruni L., Clifford G., Curado M. P., Pineros M. (2008). Burden and trends of type-specific human papillomavirus infections and related diseases in the Latin America and Caribbean region. *Vaccine*.

[11] Ciftci H. I., Can M., Ellakwa D. E. (2020). Anticancer activity of Turkish marine extracts: a purple sponge extract induces apoptosis with multitarget kinase inhibition activity. *Investigational New Drugs*.

[12] Kuruppu A. I., Paranagama P., Goonasekara C. (2019). Medicinal plants commonly used against cancer in traditional medicine formulae in Sri Lanka. *Saudi Pharmaceutical Journal*.

[13] Artun F. T., Karagoz A., Ozcan G. (2016). In vitro anticancer and cytotoxic activities of some plant extracts on HeLa and Vero cell lines. *Journal of BUON*.

[14] Akindele A. J., Wani Z., Mahajan G. (2014). Anticancer activity of *Aristolochia ringens* Vahl. (Aristolochiaceae). *Journal of Traditional and Complementary Medicine*.

[15] Dantu A. S., Shankarguru P., Ramya D. D., Vedha H. B. (2012). Evaluation of in vitro anticancer activity of hydroalcoholic extract of *Tabernaemontana divaricate*. *Asian Journal of Pharmaceutical and Clinical Research*.

[16] Efferth T., Herrmann F., Tahrani A., Wink M. (2011). Cytotoxic activity of secondary metabolites derived from Artemisia annua L. towards cancer cells in comparison to its designated active constituent artemisinin. *Phytomedicine*.

[17] Silva V. A., Alves A. L., Rosa M. N. (2019). Hexane partition from Annona crassiflora Mart. promotes cytotoxity and apoptosis on human cervical cancer cell lines. *Investigational New Drugs*.

[18] Hassan M., Watari H., AbuAlmaaty A., Ohba Y., Sakuragi N. (2014). Apoptosis and molecular targeting therapy in cancer. *BioMed Research International*.

[19] Kim R., Emi M., Tanabe K. (2014). The role of apoptosis in cancer cell survival and therapeutic outcome. *Cancer Biology and Therapy*.

[20] Jabbarzadeh Z., Khosh-Khui M. (2005). Factors affecting tissue culture of Damask rose (Rosa damascena Mill.). *Scientia Horticulturae*.

[21] Hongratanaworakit T. (2009). Relaxing effect of rose oil on humans. *Natural Product Communications*.

[22] Boskabady M. H., Shafei M. N., Saberi Z., Amini S. (2011). Pharmacological effects of Rosa damascena. *Iranian Journal of Basic Medical Sciences*.

[23] Sharafkhandy A. (1990). *Ave-Sina. Law in Medicine. Interpreter, Teheran*.

[24] Shafei M. N., Rakhshandah H., Boskabady M. H. (2003). Antitussive effect of Rosa damascena in guinea pigs. *Iranian Journal of Pharmaceutical Research*.

[25] Arezoomandan R., Kazerani H. R., Behnam-Rasooli M. (2011). The laxative and prokinetic effects of Rosa damascena Mill in rats. *Iranian Journal of Basic Medical Sciences*.

[26] Rakhshandah H., Dolati K., Hosseini M. (2008). Antinoceptive effect of Rosa damascena in mice. *Journal of Biological Sciences*.

[27] Awale S., Tohda C., Tezuka Y., Miyazaki M., Kadota S. (2011). Protective Effects of Rosa damascena and Its Active Constituent on A*β*(25–35)-Induced Neuritic Atrophy. *Evidence Based Complementary and Alternative Medicin*.

[28] Boskabady M. H., Vatanprast A., Parsee H., Ghasemzadeh M. (2011). Effect of aqueous-ethanolic extract from Rosa damascena on guinea pig isolated heart. *Iranian Journal of Basic Medical Sciences*.

[29] Kumar N., Bhandari P., Singh B., Bari S. S. (2009). Antioxidant activity and ultra-performance LC-electrospray ionization-quadrupole time-of-flight mass spectrometry for phenolics-based fingerprinting of Rose species: Rosa damascena, Rosa bourboniana and Rosa brunonii. *Food and Chemical Toxicology*.

[30] Ulusoy S., Boşgelmez-Tınaz G., Seçilmiş-Canbay H. (2009). Tocopherol, carotene, phenolic contents and antibacterial properties of rose essential oil, hydrosol and absolute. *Current Microbiology*.

[31] Mahmood N., Piacente S., Pizza C., Burke A., Khan A. I., Hay A. J. (1996). The anti-HIV activity and mechanisms of action of pure compounds isolated from *Rosa damascene*. *Biochemical and Biophysical Research Communications*.

[32] Gholamhoseinian A., Fallah H. (2009). Inhibitory effect of methanol extract of *Rosa damascena* Mill. flowers on *α*-glucosidase activity and postprandial hyperglycemia in normal and diabetic rats. *Phytomedicine*.

[33] Jafari M., Zarban A., Pham S., Wang T. (2008). R*osa damascena* decreased mortality in adult Drosophila. *Journal of Medicinal Food*.

[34] Latifi G., Ghannadi A., Minaiyan M. (2015). Anti-inflammatory effect of volatile oil and hydroalcoholic extract of Rosa damascena Mill. on acetic acid-induced colitis in rats. *Research in Pharmaceutical Sciences*.

[35] Zu Y., Yu H., Liang L. (2010). Activities of ten essential oils towards *Propionibacterium acnes* and PC-3, A-549 and MCF-7 cancer cells. *Molecules*.

[36] Zamiri-Akhlaghi A., Rakhshandeh H., Tayarani-Najaran Z., Mousavi S. H. (2011). Study of cytotoxic properties of *Rosa damascena*extract in human cervix carcinoma cell line. *Avicenna Journal of Phytomedicine*.

[37] Venkatesan B., Subramanian V., Tumala A., Vellaichamy E. (2014). Rapid synthesis of biocompatible silver nanoparticles using aqueous extract of *Rosa damascena* petals and evaluation of their anticancer activity. *Asian Pacific Journal of Tropical Medicine*.

[38] Abdel-Hameed E. S., Bazaid S. A., Hagag H. A. (2015). Chemical characterization of Rosa damascena Miller var. trigintipetala Dieck essential oil and its in vitro genotoxic and cytotoxic properties. *Journal of Essential Oil Research*.

[39] Bura F. T., Firuzja R. A., Nemati F. (2016). Cytotoxic effect of the flower and leaf bud extract of Crataegus microphylla C. Koch on HeLa cell line. *IIOAB Journal*.

[40] Al-Oqail M. M., Al-Sheddi E. S., Farshori N. N. (2019). Corn silk (Zea mays L.) induced apoptosis in human breast cancer (MCF-7) cells via the ROS-mediated mitochondrial pathway. *Oxidative Medicine and Cellular Longevity*.

[41] Lowry O. H., Rosebrough N. J., Farr A. L., Randall R. J. (1951). Protein measurement with the Folin phenol reagent. *Journal of Biological Chemistry*.

[42] Buege J. A., Aust S. D. (1978). Microsomal lipid peroxidation. *Methods in Enzymology*.

[43] Chandra D., Ramana K. V., Wang L., Christensen B. N., Bhatnagar A., Srivastava S. K. (2002). Inhibition of fiber cell globulization and hyperglycemia-induced lens opacification by aminopeptidase inhibitor bestatin. *Investigative Ophthalmology and Visual Science*.

[44] Siddiqui M. A., Kashyap M. P., Kumar V., Al-Khedhairy A. A., Musarrat J., Pant A. B. (2010). Protective potential of trans-resveratrol against 4-hydroxynonenal induced damage in PC12 cells. *Toxicology In Vitro*.

[45] Studzińska-Sroka E., Piotrowska H., Kucińska M., Murias M., Bylka W. (2016). Cytotoxic activity of physodic acid and acetone extract from Hypogymnia physodes against breast cancer cell lines. *Pharmaceutical Biology*.

[46] Mosmann T. (1983). Rapid colorimetric assay for cellular growth and survival: application to proliferation and cytotoxicity assays. *Journal of Immunological Methods*.

[47] Cudazzo G., Smart D. J., McHugh D., Vanscheeuwijck P. (2019). Lysosomotropic-related limitations of the BALB/c 3T3 cell-based neutral red uptake assay and an alternative testing approach for assessing e-liquid cytotoxicity. *Toxicology In Vitro*.

[48] Hagag H. A., Bazaid S. A., Abdel-Hameed E. S., Salman M. (2014). Cytogenetic, cytotoxic and GC–MS studies on concrete and absolute oils from Taif rose, Saudi Arabia. *Cytotechnology*.

[49] Yedjou C. G., Tchounwou P. B. (2012). In vitro assessment of oxidative stress and apoptotic mechanisms of garlic extract in the treatment of acute promyelocytic leukemia. *Journal of Cancer Science and Therapy*.

[50] Abdullah A. S., Mohammed A. S., Rasedee A., Mirghani M. E. (2015). Oxidative stress-mediated apoptosis induced by ethanolic mango seed extract in cultured estrogen receptor positive breast cancer MCF-7 cells. *International Journal of Molecular Sciences*.

[51] Al-Oqail M. M., Siddiqui M. A., Al-Sheddi E. S. (2016). V*erbesina encelioides*: cytotoxicity, cell cycle arrest, and oxidative DNA damage in human liver cancer (HepG2) cell line. *BMC Complementary and Alternative Medicine*.

[52] Kwon D. H., Cha H. J., Lee H. (2019). Protective effect of glutathione against oxidative stress-induced cytotoxicity in RAW 264.7 macrophages through activating the nuclear factor erythroid 2-related factor-2/heme oxygenase-1 pathway. *Antioxidants*.

[53] Traverso N., Ricciarelli R., Nitti M. (2013). Role of glutathione in cancer progression and chemoresistance. *Oxidative Medicine and Cellular Longevity*.

[54] Wageesha N. D., Soysa P., Atthanayake K., Choudhary M. I., Ekanayake M. (2017). A traditional poly herbal medicine “Le Pana Guliya” induces apoptosis in HepG 2 and HeLa cells but not in CC1 cells: an in vitro assessment. *Chemistry Central Journal*.

[55] Pi J., Cai H., Jin H. (2015). Qualitative and quantitative analysis of ROS-mediated oridonin-induced oesophageal cancer KYSE-150 cell apoptosis by atomic force microscopy. *PLoS One*.

[56] Tsang W. P., Chau S. P., Kong S. K., Fung K. P., Kwok T. T. (2003). Reactive oxygen species mediate doxorubicin induced p53-independent apoptosis. *Life Sciences*.

[57] González-Chavarría I., Duprat F., Roa F. J. (2020). Maytenus disticha extract and an isolated *β*-dihydroagarofuran induce mitochondrial depolarization and apoptosis in human cancer cells by increasing mitochondrial reactive oxygen species. *Biomolecules*.

[58] Jakubowicz-Gil J., Langner E., Bądziul D., Wertel I., Rzeski W. (2013). Apoptosis induction in human glioblastoma multiforme T98G cells upon temozolomide and quercetin treatment. *Tumor Biology*.

[59] Kuete V., Donfack A. R., Mbaveng A. T., Zeino M., Tane P., Efferth T. (2015). Cytotoxicity of anthraquinones from the roots of Pentas schimperi towards multi-factorial drug-resistant cancer cells. *Investigational New Drugs*.

[60] Turan I., Demir S., Kilinc K. (2018). Cytotoxic effect of Rosa canina extract on human colon cancer cells through repression of telomerase expression. *Journal of Pharmaceutical Analysis*.

[61] Kilinc K., Demir S., Turan I. (2020). Rosa canina extract has antiproliferative and proapoptotic effects on human lung and prostate cancer cells. *Nutrition and Cancer*.

[62] Wiseman D. A., Werner S. R., Crowell P. L. (2007). Cell cycle arrest by the isoprenoids perillyl alcohol, geraniol, and farnesol is mediated by p21Cip1 and p27Kip1 in human pancreatic adenocarcinoma cells. *Journal of Pharmacology and Experimental Therapeutics*.

[63] Khatib H., Rezaei-Tavirani M., Keshel S. H. (2013). Flow cytometry analysis of Rosa Damascena effects on gastric cancer cell line (MKN45). *Iranian Journal of Cancer Prevention*.

[64] Sa T., Das T. (2008). Anti cancer effects of curcumin: cycle of life and death. *Cell Division*.

